RETRACTED

# Observation of the Effect of Focused Psychological Intervention Combined with Standardized Pain Nursing on Postoperative Pain Levels and Depression and Anxiety in Patients with Intestinal Obstruction

**DOI:** 10.1155/2022/2467887

**Published:** 2022-05-04

**Authors:** Mantian Yin, Jifang Li, Jie Wang, Minxiang Li, Long Li, Genmei Wang, Yibin Ouyang, Peiru Wang

**Affiliations:** ^1^Department of Nursing, The Second Affiliated Hospital of Hainan Medical College, China; ^2^Department of General Surgery, The Second Affiliated Hospital of Hainan Medical College, China; ^3^Hainan Health Management College, China; ^4^Department of Neurosurgery, The Second Affiliated Hospital of Hainan Medical College, China; ^5^Department of Breast and Thyroid Surgery, The Second Affiliated Hospital of Hainan Medical College, China

## Abstract

**Objective:**

The purpose of this study was to investigate the effect of targeted psychological intervention combined with standardized pain care on postoperative pain, depression, and anxiety in patients with intestinal obstruction.

**Methods:**

84 patients with intestinal obstruction hospitalized at our hospital from October 2019 to February 2021 were randomly divided into study and control groups. The patients in the control group were treated with routine nursing, and the patients in the study group were treated with focused psychological intervention combined with standardized pain nursing. The pain degree (VAS), depression and anxiety (SDS, SAS) score, sleep quality (PSQI) score, and nursing satisfaction of the two groups before and after intervention were calculated.

**Results:**

Before intervention, no significant differences in VAS score between the study and control groups were observed. The VAS score of 6 h, 12 h, 24 h, and 48 h dry prognosis in the study group was lower than that in the control group. There was no significant difference in the scores of SDS and SAS between two groups. After intervention, the scores of SDS and SAS in the study group were lower than those in the control group. After intervention, the scores of daytime dysfunction, hypnotic drugs, sleep disorders, sleep efficiency, sleep time, and sleep quality in the study group were significantly lower than those in the control group. The scores of nursing state, nursing technique, nurse-patient communication, and inspection observation in the study group were higher than those in the control.

**Conclusion:**

The intervention of focused psychological intervention combined with standardized pain nursing on patients with intestinal obstruction can effectively relieve their negative emotion and reduce the degree of postoperative pain. In addition, it can improve patients' sleep quality and enhance patients' satisfaction with all kinds of nursing work.

RETRACTED

## 1. Introduction

Intestinal obstruction is mainly caused by the difficulty in expelling intestinal contents, which is a multiple acute abdomen of the digestive tract, which can cause changes in intestinal function and anatomical structure, resulting in systemic physiological disorders [1, 2]. In addition, intestinal obstruction has an acute onset and complex etiology, and patients often experience pain of varying degrees, leading to depression and anxiety and causing considerable harm to patients' physical and mental health and quality of life [3, 4]. Therefore, it is of great significance to implement effective psychological and pain interventions in the treatment of intestinal obstruction.

Psychological intervention and pain intervention have certain effects on the treatment of intestinal obstruction. However, the overall effect was different from clinical expectations. Standardized pain care and targeted psychological intervention are also commonly used clinical nursing intervention models, which play an important role in the rehabilitation of various diseases. However, there are few systematic studies on their combination in the treatment of intestinal obstruction [5–7].

This study is aimed at conducting a group study on patients with intestinal obstruction in our hospital. The purpose of this study is to clarify the application value of targeted psychological intervention combined with standardized pain care. It is expected to provide new ideas and practical reference for the nursing intervention of intestinal obstruction.

## 2. Materials and Methods

### 2.1. General Data

A total of 84 patients with intestinal obstruction was hospitalized at our hospital from October 2019 to February 2021. All patients were randomly divided into the study group (*n* = 42) and the control group (*n* = 42). There were 23 males and 19 females, aged from 38 to 64 years, with an average of 50.94 ± 11.71 years in the study group. The degree of obstruction: 13 cases of complete obstruction and 29 cases of partial obstruction. There were 26 males and 16 females, the average age was 53.01 ± 10.67 years, and the degree of obstruction was complete obstruction (*n* = 17) and partial obstruction (*n* = 25) in the control group. No significant differences were observed between the two groups (*P* > 0.05). All patients signed the consent form, and this study was approved by the Ethics Committee of our hospital.

### 2.2. Selection Criteria

Selection criteria are as follows: (1) patients who confirmed by clinical manifestations, comprehensive B-ultrasound, imaging examination, and laboratory examination; (2) age > 18 years old; (3) patients with no hematological disease; (4) patients with no malignant tumor; (5) patients with no organic lesions such as kidney and liver; (6) patients with no verbal communication disorder, cognitive dysfunction, and mental system disease; (7) exclusion of voluntary withdrawal; and (7) exclusion of patients who died during the study.

RETRACTED

### 2.3. Methods

The patients in the control group were given routine care, including parenteral nutrition support, low-flow oxygen inhalation, fasting and drinking, adjusting the infusion volume and speed to maintain water and electrolyte balance, closely monitoring the patient's vital signs, gastrointestinal decompression, and absolute bed rest. When the patient's condition is stable and physical condition allows, encourage and assist the patient to get out of bed, prevent intestinal adhesion, speed up the recovery of intestinal function, and urge the patient to strictly abide by the doctor's advice.

The patients in the study group were given targeted psychological intervention combined with standardized pain care, and on the basis of the control group, targeted psychological interventions, including (1) open psychological intervention, were introduced to the patients in detail about the treatment measures, hospitalization environment, and basic conditions of the relevant medical staff. Eliminate or relieve the patient's sense of strangeness and tension. (2) Positive psychological guidance: ercj pay close attention to the psychological dynamics of patients, encourage patients to take positive behaviors to adjust their psychological state and physical feelings, and inform patients of the beneficial effects of positive behaviors. And help them establish goals that are easily achievable during the current phase of recovery. In addition, patients are guided to recall successful experiences after solving problems during the rehabilitation process, and patients are encouraged to make continuous changes. (3) Heuristic psychological intervention: nurses actively communicate with patients, guide and encourage patients to raise their inner doubts, give patients detailed answers, and guide patients to adjust their mentality in a planned and real-time manner, to ensure that patients face the disease and related treatment with a peaceful and optimistic attitude. (4) Discuss psychological intervention, refer to the patient's psychological state and personality characteristics, discuss the treatment of the disease with the patient with a sincere attitude, and pay attention to the protection and respect of the patient's privacy during the intervention.

Standardized pain care: (1) establish a pain management team, headed by the head nurse of the department and experienced nursing staff as team members. The head nurse is responsible for formulating and coordinating nurses' work processes and responsibilities at all levels. Supervise the implementation of relevant work and find deficiencies in a timely manner. In addition, the team members were trained on pain-related knowledge, including how to assess pain and choose analgesics, physical analgesia measures, and possible adverse reactions after the use of analgesics. (2) Develop nursing intervention process with nursing evaluation-nursing diagnosis-implementation-evaluation as the basic framework, formulate corresponding pain management process, evaluate the pain degree of patients, adopt targeted intervention plan, and evaluate the intervention effect after treatment. If the effect is not good, adjust and improve. (3) Formulate a pain relief plan according to the patient's condition and degree of pain. If drug analgesia is used, the safety of the drug should be closely monitored, and the patient should be informed to strictly follow the doctor's advice, and it is strictly forbidden to increase the dose without authorization to prevent the occurrence of related adverse reactions. (4) Systematically explain pain knowledge to patients and their families, formulate pain-related knowledge manuals, ensure that patients understand the causes of pain, the significance of analgesia and its benefits to the disease, and ensure that patients can actively cooperate with analgesic interventions. (5) Evaluate and record the degree of pain in detail, comprehensively evaluate the degree of pain in the resting state and breathing state, and clarify the effect of pain on the patient's sleep.

RETRACTED

### 2.4. Observation Index

(1) The VAS scale was used to evaluate the pain degree of the two groups before the intervention and 6, 12, 4, and 48 hours after the intervention. The score ranged from 0 to 10. The higher the score, the stronger the pain [8]. (2) Statistical scores of depressions and anxiety before and after the intervention in the two groups: depression was assessed according to the SDS scale. SDS score ≥ 53 can be regarded as depression, and the higher the score, the more serious the condition. Anxiety was assessed according to the SAS scale, with a SAS score of ≥50 being considered anxiety, with higher scores indicating more seriousness [9]. (3) According to the Pittsburgh Sleep Quality Index (PSQI), the sleep quality of the two groups before and after the intervention was evaluated, including daytime dysfunction, hypnotic medication, sleep disturbance, sleep efficiency, sleep duration, and sleep quality. On a scale of 0-3, the lower the score indicated the better the sleep quality [10]. (4) Statistics on the degree of satisfaction with nursing work between the two groups, including nursing attitude, nursing skills, nurse-patient communication, inspection and observation, the score range of each dimension is 0-100 points, the higher the score, the higher the satisfaction.

RETRACTED

### 2.5. Statistical Analysis

The data were analyzed by SPSS 22.0, measurement data were expressed with (*x* ± *s*), and conducted *t*-test, counting data were expressed with *n* (%), and conducted *χ*^2^ test. The one-sided *P* < 0.05 indicated that the difference was statistically significant.

## 3. Results

### 3.1. VAS Score Comparison

As shown in Table 1, there were no significant differences of VAS score between the study group (6.56 ± 1.19) and the control group (6.81 ± 1.35) (*P* > 0.05) before intervention. The VAS scores of 6, 12, 24, and 48 dry prognosis in the study group were significantly lower than those in the control group (*P* < 0.05).

### 3.2. SDS and SAS Score

Before intervention, there were no significant differences of the scores of SDS and SAS between the study group (*P* > 0.05). After intervention, the scores of SDS and SAS in the study group (SDS, 41.61 ± 5.35; SAS, 43.39 ± 4.56) were lower than those in the control group (SDS, 45.95 ± 6.11; SAS, 48.64 ± 5.92) (*P* < 0.05, Table 2).

### 3.3. PSQI Score

As shown in Table 3, before intervention, there were no significant differences between research group of daytime dysfunction (2.22 ± 0.36), hypnotics (2.17 ± 0.61), sleep disorder (2.39 ± 0.40), sleep efficiency (2.31 ± 0.37), sleep time (2.25 ± 0.33), falling asleep time (2.37 ± 0.39), and sleep quality (2.38 ± 0.41) and control group (2.19 ± 0.40, 2.23 ± 0.57, 2.44 ± 0.45, 2.26 ± 0.40, 2.30 ± 0.29, 2.34 ± 0.42, and 2.45 ± 0.45) (*P* > 0.05). After intervention, the scores of daytime dysfunction, hypnotic drugs, sleep disorders, sleep efficiency, sleep time, sleep time, and sleep quality in the study group were 1.29 ± 0.18, 1.08 ± 0.15, 1.21 ± 0.19, 1.15 ± 0.17, 1.17 ± 0.16, 1.23 ± 0.20, and 1.30 ± 0.14, respectively, which were lower than those in the control group (1.51 ± 0.20, 1.44 ± 0.19, 1.52 ± 0.28, 1.48 ± 0.23, 1.50 ± 0.22, 1.49 ± 0.25, and 1.61 ± 0.21) (*P* < 0.05), respectively.

### 3.4. Satisfaction Degree of Nursing Work

As shown in Table 4, the scores of nursing state (96.18 ± 3.04), nursing technique (97.07 ± 2.54), nurse-patient communication (95.94 ± 4.01), and inspection observation (97.22 ± 2.37) in the study group were higher than those in the control group (92.02 ± 4.11, 93.96 ± 3.75, 90.96 ± 3.22, and 94.01 ± 3.05) (*P* < 0.05).

RETRACTED

## 4. Discussion

Intestinal obstruction is a clinical multiple acute abdomen disease with a mortality rate of about 5%-10%. Previous studies have shown that intestinal obstruction can not only cause physical harm but also lead to psychological problems such as depression and anxiety [11, 12]. Furthermore, those who lack correct recognition of intestinal obstruction lack confidence in the treatment of the disease, and the above psychological problems are more prominent [13–15]. Therefore, it is very important to implement nursing measures in a timely manner to intervene in patients with intestinal obstruction.

Focused psychological intervention is an important clinical psychological nursing model, mainly through heuristic, open, discussion, and other psychological nursing paths to regulate the psychological state of patients [16, 17]. By carrying out targeted psychological care, the daily living ability of patients with chronic renal failure can be effectively improved. In addition, patients with intestinal obstruction often have obvious pain, and pain intervention should be attached great importance to while relieving the negative emotions of patients. Standardized pain care is mainly to form an intervention group according to the specific situation of the patient. The purpose is to train the group members before nursing, improve the comprehensive nursing ability of the members, and ensure the provision of high-quality nursing services for the patients. Standardized pain care can also prevent deficiencies in nursing interventions from affecting the quality of care and provide health education to patients and their families to enhance understanding of pain-related knowledge and improve self-care capabilities. The results showed that the degree of pain was effectively relieved in all periods of time after the operation, and it could also relieve the anxiety of patients [18, 19].

Previous studies have confirmed the clinical value of targeted psychological interventions and standardized pain care. The VAS, SDS, and SAS scores of the study group were lower than those of the control group. After applying the above two measures to patients with intestinal obstruction, the PSQI score of the study group was lower than that of the control group. The results show that the intervention plan combining key psychological intervention and standardized pain care has significant advantages in reducing pain, depression, and anxiety in patients with intestinal obstruction and is also of great significance in improving the quality of sleep in patients. The main reason is that the focused psychological intervention can comprehensively intervene through heuristic, open, discussion, and other psychological nursing paths based on the detailed analysis results of the psychological problems of patients with intestinal obstruction, to adjust the negative emotions of patients and stimulate their positive emotions. Actively cooperate with nursing treatment and other related operational attitudes. Standardized pain care is a new approach to pain management. Compared with traditional nursing intervention, standardized pain care can give full play to the subjective initiative of nurses and improve the standardized level of pain care. Train nurses on basic pain knowledge and nursing programs before nursing, improve nurses' awareness of pain and nursing skills, and provide patients with targeted and effective nursing services. Bonkowski et al. [20] also pointed out that compared with routine nursing intervention, standardized pain nursing can establish a standardized pain intervention system, which can improve patients' cognitive concept of pain and change the existing mode of adverse pain management. It is of great significance to reduce the degree of postoperative anxiety. In addition, the combination of focused psychological intervention and standardized pain nursing can improve the negative mood of patients with intestinal obstruction, reduce the degree of pain, ensure that patients spend the perioperative period in good physical and mental condition, and improve their sleep quality. This method also shortens the process of postoperative rehabilitation. Our results showed that the satisfaction scores of various nursing services in the study group were higher than those in the control group, suggesting that patients with intestinal obstruction were more satisfied with targeted psychological intervention and standardized pain care. Combined intervention programs can more effectively improve patients' physical and mental status and sleep quality. In addition, it is helpful to reduce nurse-patient disputes and establish a good service image.

RETRACTED

In conclusion, targeted psychological intervention combined with standardized pain nursing intervention for patients with intestinal obstruction can effectively relieve patients' negative emotions, reduce postoperative pain, improve patients' sleep quality, and enhance patients' satisfaction with various nursing work.

## Figures and Tables

**Table 1:** Comparison of VAS scores between the two groups ($\bar{x}\pm s$).

Group	Number	Before intervention	6 hours after intervention	12 hours after intervention	24 hours after intervention	48 hours after intervention
Research group	42	6.56 ± 1.19	2.41 ± 1.01	1.89 ± 0.69	2.04 ± 0.75	2.01 ± 0.80
Control group	42	6.81 ± 1.35	4.63 ± 1.24	3.04 ± 0.83	3.15 ± 0.93	2.94 ± 0.96
*t*		0.900	8.996	6.905	6.021	4.823
*P*		0.371	<0.001	<0.001	<0.001	<0.001

**Table 2:** Comparison of SDS and SAS scores between the two groups ($\bar{x}\pm s$).

Time	Group	Number	SAS	SDS
Before intervention	Research group	42	62.32 ± 5.67	60.67 ± 5.96
	Control group	42	60.98 ± 6.11	61.79 ± 6.37
	*t*		1.042	0.832
	*P*		0.301	0.408
After intervention	Research group	42	43.39 ± 4.56	41.61 ± 5.35
	Control group	42	48.64 ± 5.92	45.95 ± 6.11
	*t*		4.553	3.463
	*P*		<0.001	0.001

**Table 3:** Comparison of PSQI scores between the two groups ($\bar{x}\pm s$).

Time	Group	Number	Daytime dysfunction	Hypnotic drug	Sleep disorder	Sleep efficiency	Sleep time	Sleeping time	Sleep quality
Before intervention	Research group	42	2.22 ± 0.36	2.17 ± 0.61	2.39 ± 0.40	2.31 ± 0.37	2.25 ± 0.33	2.37 ± 0.39	2.38 ± 0.41
	Control group	42	2.19 ± 0.40	2.23 ± 0.57	2.44 ± 0.45	2.26 ± 0.40	2.30 ± 0.29	2.34 ± 0.42	2.45 ± 0.45
	*t*		0.361	0.466	0.538	0.595	0.738	0.339	0.745
	*P*		0.719	0.643	0.592	0.554	0.463	0.735	0.458
After intervention	Research group	42	1.29 ± 0.18	1.08 ± 0.15	1.21 ± 0.19	1.15 ± 0.17	1.17 ± 0.16	1.23 ± 0.20	1.30 ± 0.14
	Control group	42	1.51 ± 0.20	1.44 ± 0.19	1.52 ± 0.28	1.48 ± 0.23	1.50 ± 0.22	1.49 ± 0.25	1.61 ± 0.21
	*t*		5.299	9.638	5.937	7.478	7.862	4.149	7.960
	*P*		<0.001	<0.001	<0.001	<0.001	<0.001	<0.001	<0.001

**Table 4:** Comparison of nursing satisfaction between the two groups ($\bar{x}\pm s$).

Group	Number	Nursing attitude	Nursing technique	Nurse-patient communication	Inspection and observation
Research group	42	96.18 ± 3.04	97.07 ± 2.54	95.94 ± 4.01	97.22 ± 2.37
Control group	42	92.02 ± 4.11	93.96 ± 3.75	90.96 ± 3.22	94.01 ± 3.05
*t*		5.274	4.450	6.276	5.386
*P*		<0.001	<0.001	<0.001	<0.001

## Data Availability

The authors confirm that the data supporting the findings of this study are available within the article.
